The article "Intelligent Monitoring System Based on Noise-Assisted Multivariate Empirical Mode Decomposition Feature Extraction and Neural Networks" was published in 2022. Journal: Comput Intell Neurosci.

# Intelligent Monitoring System Based on Noise-Assisted Multivariate Empirical Mode Decomposition Feature Extraction and Neural Networks

**DOI:** 10.1155/2022/2698498

**Published:** 2022-04-25

**Authors:** Le Fa Zhao, Shahin Siahpour, Mohammad Reza Haeri Yazdi, Moosa Ayati, Tian Yu Zhao

**Affiliations:** ^1^School of General Education, Shenyang Sport University, Shenyang 110115, China; ^2^Department of Mechanical Engineering, University of Cincinnati, Cincinnati 45221, USA; ^3^School of Mechanical Engineering, University of Tehran, Tehran, Iran; ^4^Key Laboratory of Structural Dynamics of Liaoning Province, College of Sciences, Northeastern University, Shenyang 110819, China

## Abstract

Because of the nonlinearity and nonstationarity in the vibration signals of some rotating machinery, the analysis of these signals using conventional time- or frequency-domain methods has some drawbacks, and the results can be misleading. In this paper, a couple of features derived from multivariate empirical mode decomposition (MEMD) are introduced, which overcomes the shortcomings of the traditional features. A wind turbine gearbox and its bearings are investigated as rotating machinery. In this method, two types of feature structures are extracted from the decomposed signals resulting from the MEMD algorithm, called intrinsic mode function (IMF). The first type of feature vector element is the energy moment of effective IMFs. The other type of vector elements is amplitudes of a signal spectrum at the characteristic frequencies. A correlation factor is used to detect effective IMFs and eliminate the redundant IMFs. Since the basic MEMD algorithm is sensitive to noise, a noise-assisted extension of MEMD, NA-MEMD, is exploited to reduce the effect of noise on the output results. The capability of the proposed feature vector in health condition monitoring of the system is evaluated and compared with traditional features by using a discrimination factor. The proposed feature vector is utilized in the input layer of the classical three-layer backpropagation neural network. The results confirm that these features are appropriate for intelligent fault detection of complex rotating machinery and can diagnose the occurrence of early faults.

## 1. Introduction

With the advent of new era of Industry 4.0, the human and machine interaction has dramatically changed [1]. The improvement and advancement in intelligent systems have paved the way for the better use of smart devices. This shifts traditional human-machine interactions (HMI) toward intelligent human-machine interactions. The application of intelligent HMI ranges from medical scenarios to industrial applications [2–5] (e.g., robotics, energy, maintenance, and semiconductor manufacturing). Among the key drivers of the transition from traditional to intelligent HMI, progress in machine learning and intelligent algorithms constitutes the main portion of importance [6–9].

The article "Intelligent Monitoring System Based on Noise-Assisted Multivariate Empirical Mode Decomposition Feature Extraction and Neural Networks" was published in 2022. Journal: Comput Intell Neurosci.

Monitoring the condition of rotating machinery plays an important role in the engineering industries [10, 11]. To detect early faults and fully inspect the health condition of rotating systems, a condition monitoring structure is required to operate as soon as possible [12, 13]. The main objective of exploiting condition monitoring systems is to improve accuracy by lowering costs. The extraction of fault characteristics from these types of systems is a key step in the process of fault detection and condition monitoring [14].

Signals from complex rotating machinery are usually nonstationary and nonlinear, and extracting features that lead to a desirable outcome has become a challenging process. Features are the parameters that are derived from signals to indicate the characteristics of systems. So far, various features that can be extracted from vibration signals have been investigated [15–17]. Signal processing to extract fault features is divided into three main domains: time domain, frequency domain, and time-frequency domain. Some conventional time-domain methods are skewness and kurtosis [18] or root mean square (RMS) and peak value of a signal [19]. Frequency analysis mostly contains Fourier spectra of a time series signal, cepstrum analysis, or envelope analysis [20, 21]. These features are in the time or frequency domain and are mostly extracted from raw vibration signals. In the presence of nonlinearity and nonstationarity in the signal, traditional features cannot have an accurate distinction between system conditions [22]. Because of these problems, time-frequency analysis of complex signals is introduced as an application of feature extraction. Time-frequency methods, such as the short-time Fourier transform [23], wavelet transform [24], empirical mode decomposition (EMD) [25], or Wigner–Ville [26], analyze signals in both time and frequency domains. Therefore, features can contain more comprehensive information of signals.

With the advent of a new time-frequency method, named Hilbert–Huang transform (HHT) [27], many studies have been conducted using this method in the field of signal processing [28–30]. HHT is a powerful algorithm useful for nonlinear and nonstationary signals, performing an adaptive decomposition operation called empirical mode decomposition (EMD). The decomposed signals, named intrinsic mode functions (IMFs), are almost monocomponents which satisfy Hilbert transform terms. Each IMF covers a small range of frequency scales. This characteristic of IMFs makes them a suitable tool for the analysis of complex systems. EMD algorithm is sensitive to noise. When signals are noisy, the mode-mixing phenomenon can occur in IMFs [31]. In this situation, either a single IMF carries a signal of a widely disparate scale, or a single mode (or scaling) exists in more than one IMF. To overcome this phenomenon, Ensemble EMD (EEMD) is proposed [32].

The article "Intelligent Monitoring System Based on Noise-Assisted Multivariate Empirical Mode Decomposition Feature Extraction and Neural Networks" was published in 2022. Journal: Comput Intell Neurosci.

When the system contains many components and has comprehensive information from all over the system, multiple sensors are located on different parts of the system. In this condition, the signals obtained from the sensors are a kind of multivariate signals. If the EMD algorithm is used on each signal individually, joint information will be wasted [33]. Furthermore, the same group of IMFs may have different characteristic information [34]. To overcome these problems, Riling et al. [35] proposed bivariate EMD. In this method, by mapping the bivariate signal in different directions, the local mean of the signal is calculated. To continue this idea, in 2010, Rehman and Mandic [36] proposed an empirical mode decomposition algorithm for trivariate signals. After that, they proposed an extension to their method and introduced multivariate EMD (MEMD) to deal with multidimensional signals [37]. This method allows us to analyze multidimensional signals simultaneously and covers the problem of using the EMD method for these kinds of signals. Zhao et al. [38] employ multivariate EMD method to extract some health condition information of the studied system. In their study, they used full spectrum based condition monitoring for rotating machinery. Lv et al. [33] used multivariate EMD as an application to investigate the health conditions of the patients.

Each IMF order resulting from the MEMD algorithm has the same frequency characteristic. This capability makes the MEMD algorithm a suitable method for feature extraction to diagnose faults in rotating systems. Some of the IMFs are spurious and need to be eliminated from the calculation to speed up the process of feature extraction and make the feature vector smaller without losing accuracy. Some IMFs are high-frequency ones, which can be regarded as noisy IMFs. In contrast, some IMFs contain low-frequency characteristics that exist due to the stopping criteria of the EMD algorithm and do not have physical meaning. Effective IMFs can be detected by user experience, but to make the process faster, a criterion or factor must be used. Ricci et al. [39] introduced a merit index that automatically selects the effective IMFs and eliminates the spurious ones. This index is based on the symmetrical and periodic IMF specifications. In [38], a sensitivity factor which is based on mutual information is proposed. In [33], a correlation factor is introduced to detect the most effective IMFs and, as is obvious from the name of the factor, it is based on the correlation between the signal and each IMF.

The article "Intelligent Monitoring System Based on Noise-Assisted Multivariate Empirical Mode Decomposition Feature Extraction and Neural Networks" was published in 2022. Journal: Comput Intell Neurosci.

The features derived from the signals can be implemented as input for an artificial neural network (ANN) system [40] or can be used for a support vector machine (SVM) [41] to analyze the conditions of the system intelligently and automatically. Yang et al. [42] extract bearing health characteristics using the energy of decomposed IMFs. They compare the output results from a simple ANN while the features are derived from wavelet analysis. Bin et al. [43] used a combined method of wavelet packet decomposition (WPD) and EMD to extract fault features from a bearing mechanism as rotating machinery. In their study, the energy moment from the IMFs is used as the feature vector. WPD is used to denoise and preprocess a signal.

To address the aforementioned issues and challenges, an intelligent feature extraction is proposed. The following are the main novelties and contributions of this study:

- The NA-MEMD algorithm is used as a feature extraction method.
- Correlation analysis is used to detect effective IMFs.
- In addition to the energy moment of effective IMFs, an amplitude factor in the frequency domain is introduced as a complementary element for the feature vector.
- To show the capability of the proposed features in the diagnosis of system conditions, a discrimination criterion is exploited to make the comparison tangible. Features are then used for a backpropagation (BP) neural network input layer.
- The proposed algorithm can be used for analyzing the features of the data from the athletes and the fault analysis of the key mechanical components in the sport field. This paper focuses on the analysis of bearings used in the key components in the sport field.

This paper is organized as follows. In Section 2, the proposed signal processing and feature extraction procedure are explained.  Section 3 is dedicated to the structure and design configuration of the neural network. In Section 4, the rotation system is introduced. In Section 5, the implementation of the proposed method on the studied system is investigated, and the results are discussed. The conclusion is presented in Section 6.

## 2. Feature Extraction Using Multivariate EMD

### 2.1. Fundamentals of Multivariate EMD

In standard EMD [27], the local mean can be calculated by interpolating the upper and lower envelope of a univariate signal. However, when dealing with multivariate signals, it is rather confusing to determine IMFs, because the value of local minima and maxima cannot be directly defined. Rehman and Mandic [37] introduce a multivariate EMD algorithm to overcome these issues. In this method, multivariate (*n*-variate) signals are considered as *n*-dimensional time series. Some appropriate direction vectors are chosen, and multivariate signals are projected on the selected direction vectors. All envelopes of these projected signals are calculated, and by averaging the envelopes, the local mean of the multivariate signal is determined. Therefore, the sifting process [31] (which is used in standard EMD) can be implemented to calculate IMF groups.

The article "Intelligent Monitoring System Based on Noise-Assisted Multivariate Empirical Mode Decomposition Feature Extraction and Neural Networks" was published in 2022. Journal: Comput Intell Neurosci.

The process of local mean calculation can be considered as an approximation of the integral of all envelopes along with the multiple directions in the *n*-dimensional space. The accuracy of this calculation depends on the uniformity of the chosen direction vectors. To generate a set of uniformly distributed points, quasi-Monte Carlo-based low-discrepancy sequences can be utilized. The Halton sequence family is exploited as a convenient way to generate a low-discrepancy sequence.

Let *x*_1_,…, *x*_*n*_ be the first *n* prime numbers, and the *i*th sample of a one-dimensional Halton sequence, denoted by *r*_*i*_^*x*^, is given by

(1) $$\begin{array}{c} r_{i}^{x}=\frac{a_{0}}{x}+\frac{a_{1}}{x^{2}}+\ldots +\frac{a_{s}}{x^{s+1}}, \end{array}$$

where the base-*x* representation of *i* is given by

(2) $$\begin{array}{c} i=a_{0}+a_{1}x+\ldots +a_{s}x^{s}\text{.} \end{array}$$

Starting from *i*=0, the *i*th sample of Halton sequence then becomes

(3) $$\begin{array}{c} \left(r_{i}^{x_{1}},r_{i}^{x_{2}},\ldots ,r_{i}^{x_{n}}\right)\text{.} \end{array}$$

The Hammersley sequence is used when the total number of samples, *n*, is known a priori; in this case, the *i*th sample within the Hammersley sequence is calculated as

(4) $$\begin{array}{c} \left(\frac{i}{n},r_{i}^{x_{1}},r_{i}^{x_{2}},\ldots ,r_{i}^{x_{n-1}}\right)\text{.} \end{array}$$

By using Halton and Hammersley sequences, a suitable set of direction vectors on the *n*-sphere is generated. Henceforth, projections of signals on this direction vector will be calculated. In the following paragraph, multivariate EMD will be explained briefly.

Let *X*(*t*)=[*x*_1_(*t*), *x*_2_(*t*),…, *x*_*n*_(*t*)] be an *n*-dimensional signal and *D*^*k*^={*d*_1_^*k*^, *d*_2_^*k*^,…, *d*_*n*_^*k*^} correspond to the *k*th direction vector in a direction set *D*. The multivariate EMD algorithm is described as follows:

(1) Choose a suitable set of direction vectors, *D*.
(2) Calculate the *k*th projection, *p*^*k*^(*t*) of *X* along the *k*th direction, where *k*=1,2,…, *K* and *K* is a total number of direction vectors.
(3) Find the time instants, *t*_*i*_^*k*^, corresponding to the maxima of projected signals.
(4) Interpolate [*t*_*i*_^*k*^, *X*(*t*_*i*_^*k*^)] to determine multidimensional envelopes, *E*^*k*^(*t*).
(5) Calculate the mean by
  (5) $$\begin{array}{c} M\left(t\right)=\frac{1}{l}\sum_{k=0}^{K}E^{k}\left(t\right)\text{.} \end{array}$$
(6) Calculate the residual component *R*(*t*) = *X*(*t*) − *M*(*t*). If *D*(*t*) satisfies the stopping criterion explained in the previous section, then consider *R*(*t*) as an IMF and then repeat the algorithm until it meets the criterion.

The article "Intelligent Monitoring System Based on Noise-Assisted Multivariate Empirical Mode Decomposition Feature Extraction and Neural Networks" was published in 2022. Journal: Comput Intell Neurosci.

### 2.2. Effect of Noise on IMFs

EMD method is sensitive to noise. In [44], an investigation is conducted on the sensitivity of MEMD to noise. It can be inferred from this study that the MEMD algorithm is sensitive to noise and mode-mixing problems that can happen in this method. An extension to MEMD is proposed to cover the problem. The extension is named noise-assisted multivariate empirical mode decomposition (NA-MEMD). NA-MEMD algorithm tries to eliminate noise interference in EEMD and reduce mode mixing in EMD and MEMD methods. The general algorithm in NA-MEMD is the same as in MEMD. The difference is that the input multivariate signal consists of input data and noise in separate channels. After the implementation of the MEMD algorithm on the new multivariate signal, the resulting noise-related IMFs will be discarded. This method is demonstrated briefly as follows:

1. Construct *l*-channel of uncorrelated Gaussian white noise time series which have the same length as that of the input (*l* ≥ 1).
2. Add noise channels, created in the previous step, to the input signals; therefore, the new input signal is (*n* + *l*)-channel.
3. Process the (*n* + *l*)-channel multivariate signal using MEMD algorithm to obtain IMFs.
4. Discard *l*-channels corresponding to the noise from (*n* + *l*)-variate IMFs and get *n*-channel IMFs corresponding to the original signal.

### 2.3. The Criterion for Choosing IMFs

To extract fault features from the signal, suitable IMFs must be selected. A suitable IMF is an IMF which has a meaningful frequency scale. The choice of IMF is usually based on experience and is done manually. This process is slow and time-consuming. To make this procedure faster and relatively automatic, an index or coefficient is needed to be introduced. One way to determine the suitability of an IMF is to calculate the correlation between the IMF and the original signal [45]. The IMF, which has a small correlation coefficient, is regarded as a redundant or noise component. With the help of the correlation coefficient, it is possible to accurately determine and eliminate the noise component and evaluate the effective IMFs to extract fault features from them.

The article "Intelligent Monitoring System Based on Noise-Assisted Multivariate Empirical Mode Decomposition Feature Extraction and Neural Networks" was published in 2022. Journal: Comput Intell Neurosci.

In dealing with the MEMD algorithm, the resulting IMFs are a set of IMF groups, and some calculation must be done to identify the effective IMFs. Hence, a fault correlation factor (FCF) has been proposed [33] to conduct the analysis. Suppose that the input signal is *n*-variate signal and there exist *n* groups for *m*th IMFs corresponding to each signal. The multivariate signal can be organized as a matrix as follows:

(6) $$\begin{array}{c} S\left(t\right)=\left[S_{1}\left(t\right),S_{2}\left(t\right),\ldots ,S_{n}\left(t\right)\right]. \end{array}$$

The *k*th IMF on *n* groups corresponds to each input signal and constitutes a matrix in the form of

(7) $$\begin{array}{c} C\left(t\right)=\left[c_{1}^{k}\left(t\right),c_{2}^{k}\left(t\right),\ldots ,c_{n}^{k}\left(t\right)\right]. \end{array}$$

A simplified form of the correlation coefficient is as follows:

(8) $$\begin{array}{c} \lambda_{xy}=\frac{\sum_{n=1}^{N}x\left(t\right)c\left(t\right)}{\sqrt{\sum_{n=1}^{N}x^{2}\left(t\right)\sum_{n=1}^{N}c^{2}\left(t\right)}}\text{,} \end{array}$$

where *t* is the time and *N* is the total number of sampling points. *λ*_*i*_^*k*^ is defined as the FCF of *i*th IMF of *C*(*t*) (7) and can be calculated by conducting correlation analysis on this IMF with each *n*-variate signal, respectively, and averaging all correlation factors. *λ*_*i*_^*k*^ indicates the correlation between this IMF and the original signal. To make a comparison between each order of IMFs, the FCF of IMFs with the same order must be calculated. It can be achieved by averaging all vector correlations since each order of IMFs contains almost the same features.

(9) $$\begin{array}{c} \lambda^{k}=\sum_{i=1}^{n}\frac{\lambda_{i}^{k}}{n}. \end{array}$$

When the value of *λ*^*k*^ is large, it means that the degree of correlation of the fault characteristic between the *k*th order IMF of the *n* IMF groups and the original signal is higher. Based on the criterion of Pearson Correlation Coefficients, when the value of the correlation coefficient is higher than 0.3, it can be assumed that the signals are relevant. Therefore with this approach, effective IMFs can be determined.

### 2.4. Feature Selection

The idea of extracting features for the diagnosis of rotating machinery faults is a critical task. Features must be selected wisely, because some features may be futile in extracting fault characteristics of a signal, although these parameters are useful for other vibration signals. To choose the most effective features, a scientific criterion, which relates the features to the system condition, can be used. To achieve this purpose, in this paper, a discrimination criterion, denoted as *J*, is applied [46]. This criterion is based on the ratio between inter- and intra-variance. Suppose *N* features are extracted for a vibration signal with *K* class of system conditions. If *r*_*k*,*n*_ is the *n*th feature of the *k*th class, the intraclass and interclass variance matrix of the average dispersion coefficients are given as follows:

(10) $$\begin{array}{c} S_{\text{intra}}=\frac{1}{K\times N}\sum_{k=1}^{K}\sum_{n=1}^{N}\left({\underline{r}}_{k,n}-{\underline{\mu }}_{k}\right){\left({\underline{r}}_{k,n}-{\underline{\mu }}_{k}\right)}^{t},\\ S_{\text{inter}}=\frac{1}{K}\sum_{k=1}^{K}\sum_{n=1}^{N}\left({\underline{r}}_{k}-{\underline{\mu }}_{c}\right){\left({\underline{r}}_{k}-{\underline{\mu }}_{c}\left(\right)\right)}^{t}, \end{array}$$

while the mean of feature vectors of the *k*th class is defined by ${\underline{\mu }}_{k}=\left(1/N\right)\sum_{n=1}^{N}{\underline{r}}_{k,n}$ and the total mean of feature vectors of all classes is ${\underline{\mu }}_{c}=\left(1/N\right)\sum_{k=1}^{K}{\underline{\mu }}_{k}$.

The article "Intelligent Monitoring System Based on Noise-Assisted Multivariate Empirical Mode Decomposition Feature Extraction and Neural Networks" was published in 2022. Journal: Comput Intell Neurosci.

Finally, *J* is computed as follows:

(11) $$\begin{array}{c} J=\text{trace}\left(S_{\text{intra}}^{-1}S_{\text{inter}}\right)\text{.} \end{array}$$

According to the criterion, for the features with a high value of *J*, the effect of the corresponding feature on the diagnosis of a specific fault becomes greater.

### 2.5. Traditional Features

Traditional fault features are simple and can easily be implemented in signals [47]. In Table 1, some of these traditional features are represented in the frequency and time domain. When a fault occurs in the rotating machinery, the time-domain signal may change both its amplitude and distribution. Moreover, the frequency spectrum may encounter some deviation from the normal condition. Usually, with the help of these features, some faults can be determined in the system.Note. *x*_*n*_ is vibration signal with *n*=1,…, *N*; *N* is the number of data points; *s*_*k*_ is the frequency spectrum of *x*_*n*_; *K* is number of spectral lines; and *f*_*k*_ is frequency value of *k*th spectral line.

### 2.6. Feature Extraction from Decomposed IMFs

In addition to the traditional features mentioned earlier, the MEMD algorithm is used to extract some other features to form a more reliable and almost more robust feature vector.

Standard EMD is designed to process univariate signals. When signals from multiple sensors (or conditions) are individually processed by the EMD algorithm, there might be two main drawbacks in the results. The first drawback is the loss of joint information. The main reason for collecting information from multiple sensors (or conditions) is to have a more comprehensive understanding of the system. By implementation of EMD algorithm individually on each signal, the idea of multiple sensors would be vain. The second drawback is about the features of the same order of IMFs in each signal. IMFs in the same order corresponding to each signal that resulted from the EMD algorithm may have different features [34]. This makes it difficult to determine the effective IMFs.

The article "Intelligent Monitoring System Based on Noise-Assisted Multivariate Empirical Mode Decomposition Feature Extraction and Neural Networks" was published in 2022. Journal: Comput Intell Neurosci.

MEMD algorithm overcomes these two problems. The IMFs, resulting from the MEMD algorithm, not only contain comprehensive information about the system, but also, in the same order of IMFs, almost consist of the same feature information. These two advantages of MEMD, in addition to the benefits of the EMD method, make this algorithm an ideal choice for extracting features contributing to multivariate signals.

As was mentioned before, each order of IMFs calculated by noise-assisted MEMD contains a small frequency scale. This characteristic paves the way for analysis and feature extraction in the frequency domain for each order of IMFs. When a fault occurs in a rotating component of a system, a natural frequency (or meshing frequency for contacting components, e.g., gearboxes) is excited, which results in a burst of energy at this frequency. To identify the fault, it is necessary to detect the frequency occurrence of these high-energy bursts. Since each IMF order is composed of a small range of frequencies, by performing frequency-domain analysis, the amplitude of the signal in characteristic frequencies can be determined. FCF is a suitable index to eliminate redundant IMFs or specifically redundant frequency bands. This amplitude can be regarded as a fault feature for implementation in smart analysis.

To clarify what was mentioned above, the procedure is implemented on the synthetic signal. The multivariate synthetic signal is given as follows:

(12) $$\begin{array}{c} x_{1}=\sin\left(2\pi f_{1}t\right)+0.5\;\cos\left(2\pi f_{2}t\right)+0.9\;\sin\left(2\pi f_{3}t\right),\\ x_{2}=0.7\;\sin\left(2\pi f_{1}t\right)+\cos\left(2\pi f_{2}t\right)+0.4\;\cos\left(2\pi f_{2}t\right),\\ x_{3}=0.9\;\sin\left(2\pi f_{1}t\right)+0.6\;\cos\left(2\pi f_{2}t\right)+\cos\left(2\pi f_{2}t\right), \end{array}$$

where *f*_1_=20 Hz, *f*_2_=50 Hz, and *f*_3_=90 Hz. The sampling point is *N*=1000, and the sampling frequency is *f*_*s*_=1000 Hz. White Gaussian noise is added to each signal. Noise signals are white Gaussian signals and the corresponding power is −10 dBW.

Since noise is added to the multivariate signal, to prevent the phenomenon of mode mixing, the NA-MEMD algorithm is implemented.  Figure 1 shows the calculated IMFs by using NA-MEMD. From this figure, it is verified that each order of IMFs has the same frequency characteristics. IMF3 to IMF5 consist of the main frequencies of component signals. The remaining IMFs are redundant ones, either high-frequency IMFs which are regarded as noise or low-frequency IMFs which are due to the stopping criterion and do not have physical meaning.

The article "Intelligent Monitoring System Based on Noise-Assisted Multivariate Empirical Mode Decomposition Feature Extraction and Neural Networks" was published in 2022. Journal: Comput Intell Neurosci.

FCF is used to determine effective IMFs and to detect which IMFs contain frequency features. In Table 2 the calculated results for FCF are shown. According to the criterion of Pearson Correlation Coefficients, since IMF3 to IMF5 have FCF higher than 0.3, they can be assumed to be relevant IMFs, which is acceptable for the manual estimation of these IMFs. Therefore, the process of selecting suitable IMFs converts to a relatively automatic procedure.

The amplitude of frequency spectrum of IMFs in characteristic frequencies is an ideal feature for fault detection of rotating machinery. In the dominant IMFs in the studied synthetic signal, there exist peaks in the propinquity of characteristic frequencies. The amplitude of these peaks is going to be used as a feature for the input of an artificial neural network, because the amplitude of these peaks changes when the system operates under different conditions. Therefore, this characteristic can make a distinction for different health conditions in the system.

To have accurate and reliable results from the neural network, features as the input of the neural network must contain the detailed information of the studied system. Vibration signals from rotating machinery are usually nonlinear and nonstationary. This specification of vibration signal, which changes the energy of the signal, is in some frequency bands. IMF components contain information corresponding to a frequency band; thus, the IMF energy can be used to characterize a signal. Instead of using energy [42] or the energy entropy of the signal [16], the energy moment [43] is used as part of the proposed characteristic vector. In this method, the time feature is used for the calculation of energy; thus, it can be a complementary feature extraction method in addition to the proposed frequency-domain method. The energy moment can distinguish signal features more accurately compared to the classical energy method when the signal is nonlinear or nonstationary, which will be explained in the following paragraphs.

The energy moment for each IMF can be calculated as

(13) $$\begin{array}{c} E_{i}=\int t.{\left|c_{i}\left(t\right)\right|}^{2}dt\text{,} \end{array}$$

and for continuous calculation and discrete analysis,

(14) $$\begin{array}{c} E_{i}=\sum_{k=1}^{n}\left(k\Delta t\right){\left|c_{i}\left(k.\Delta t\right)\right|}^{2}, \end{array}$$

where *n* is the total number of sampling points, Δ*t* is the period of samples, and *k* is the number of the sample points.

The article "Intelligent Monitoring System Based on Noise-Assisted Multivariate Empirical Mode Decomposition Feature Extraction and Neural Networks" was published in 2022. Journal: Comput Intell Neurosci.

Energy moment can form a feature vector as follows:

(15) $$\begin{array}{c} T=\left[E_{1},E_{2},\ldots ,E_{n}\right]. \end{array}$$

Because the energy moment has a high value, *T* can be adjusted using normalization. Assume *E*=∑_*i*=1_^*n*^*E*_*i*_; then,

(16) $$\begin{array}{c} T_{n}=\left[\frac{E_{1}}{E},\frac{E_{2}}{E},\ldots ,\frac{E_{n}}{E}\right], \end{array}$$

where *T*_*i*_ is normalized energy moment for signal *c*_*i*_. As is clear from (13) and (14), the moment energy contains both the signal energy and the signal distribution in the time domain (because of the term *t* in the equations), indicating the advantage of the moment energy over the calculation of the classical energy [43].

## 3. Neural Network Structure

A BP neural network is designed to intelligently diagnose faults in rotating machinery. To do so, a neural model of BP must be structured. A typical BP neural network structure is illustrated in Figure 2. This network has one hidden layer. In the field of rotating machinery fault detection, the input layer contains features extracted from the original signal, and the output layer is the system health conditions (i.e., being healthy or having a specific fault type).

The number of hidden layer cells cannot be defined accurately. If the hidden layer nodes are too high, the connection between nodes increases, and as a result, the number of connection weights increases, making the neural network training process more complex. If the hidden layer nodes are too small, the accuracy of the output results cannot be guaranteed. For a three-layer network (one hidden layer), there is an empirical and experimental relationship that relates the number of hidden layer nodes *k* to the number of input layer nodes *n* [43]. The relationship is given as follows:

(17) $$\begin{array}{c} k=2n+i,0\leq i\leq 8. \end{array}$$

Note that even in this relationship, *k* is not definite and can be changed.

In Figure 3, an overview of smart fault detection of rotating machinery is illustrated schematically.

## 4. System Description

To explain the proposed method, this paper investigates the transmission system in the wind turbine system (gearbox and bearing), as a rotating machinery. The vibration data from the experiment were provided by the National Renewable Energy Laboratory (NREL). The system is depicted in Figure 4. As is indicated in the figure, the main sections rotate at the three speed stages, i.e., the low-speed stage (LSS), the intermediate-speed stage (ISS), and the high-speed stage (HSS). The test drive is designed for the wind turbine with rated power of 750 kW. The overall ratio for the gearbox system is 1 : 81.491. In Table 3, more details on the description of the gearbox are shown [48].

The article "Intelligent Monitoring System Based on Noise-Assisted Multivariate Empirical Mode Decomposition Feature Extraction and Neural Networks" was published in 2022. Journal: Comput Intell Neurosci.

To obtain vibration data from the gearbox system, accelerometers are mounted on the top of the gearbox. Data are collected at a rate of 40 kHz per channel using a National Instruments PXI-4472B high-speed data acquisition system (DAQ). Eight sensors are located in different places of the system to obtain comprehensive information from the gearbox system.

As was mentioned in the previous section, the feature vectors contain some components which are related to the amplitude of the frequency spectrum with the characteristic frequency. Characteristic frequency encompasses not only the rotating frequencies of the components but also the meshing frequencies of linked components. The studied system in faulty condition corresponds to three major fault types. The formulation for the calculation of the main characteristic frequencies is briefly illustrated in Table 4.

For the gearbox of fixed axis, *f*_1_, *f*_2_, *N*_1_, and *N*_2_ are the frequency of the pinion, the frequency of the gear, the number of teeth in the pinion, and the number of teeth in the gear, respectively. For the planetary stage, *f*_*s*_, *N*_*s*_, *N*_*R*_, and *N*_*p*_ are the sun frequency, the number of suns, the ring gear, and the teeth of the planet, respectively. For the bearing, *f*_*r*_, *n*, *ϕ*, *d*, and *D* are the shaft speed, the number of rolling elements, the angle of the load from the radial plane, the rolling element diameter, and the bearing average diameter, respectively. In Figure 5, the main dominant characteristic frequencies are shown schematically. These frequencies are high-speed shaft (HSS) frequency, planetary gear mesh frequency (PLTGM), high-speed shaft bearing B (Figure 4), high-speed shaft gear mesh (HSGM), and its second and third harmonics.

## 5. Method Implementation on System and Discussion

### 5.1. Feature Extraction for the System

As was mentioned, the input layer in the neural network is a vector constructed from fault features. Some elements are composed of normalized energy moments. First, a windowing process is implemented on the input signal to construct as many signals as possible for the input of the NA-MEMD algorithm as the input of the neural network. The signals provided by NREL are made up of 10 signals of 60 s duration. Each signal contains 2400000 data samples. A window is a section of each signal with 240000 data samples without overlapping which divides the corresponding signal into 10 subsignals. Thus, for each condition of the system, 100 features can be constructed. Windowing increases the feature vectors, increasing the accuracy of neural network operation. Subsections are now considered as input to the MEMD algorithm to obtain IMFs. To avoid the mode-mixing phenomenon, NA-MEMD is used instead of the MEMD algorithm. 3 white Gaussian noises with a variance of 0.1 are added as 3 new channels to the multivariate input signal. In Figure 6, the resulting IMFs for one channel of the multivariate faulty signal are shown. 20 IMFs are extracted from the NA-MEMD while some of them are spurious and must be omitted from the consideration. In Table 5, FCF values calculated for the IMFs are shown. IMFs of orders three to eight have an FCF higher than 0.3; thus, these IMF groups are considered as effective IMFs for the calculation of energy moment.

The article "Intelligent Monitoring System Based on Noise-Assisted Multivariate Empirical Mode Decomposition Feature Extraction and Neural Networks" was published in 2022. Journal: Comput Intell Neurosci.

The feature selection algorithm is applied to the proposed features. For the system studied, two classes of system conditions are considered (*K*=2) and 30 characteristics are extracted (*N* = 30). The resultant discrimination criterion is shown in Table 6. According to the table, the values of *J* for most of the MEMD characteristics are greater than the traditional characteristics except for the value of *pt*_1_ (that is, the root mean square). This shows that the proposed features can be suitable for detecting faults in the wind turbine gearbox studied. Therefore, the feature vector can be constructed as follows:

(18) $$\begin{array}{c} F=\left[E_{3}^{\prime },E_{4}^{\prime },E_{5}^{\prime },E_{6}^{\prime },E_{7}^{\prime },E_{8}^{\prime },AF_{6},AF_{8},AF_{11}\right]\text{,} \end{array}$$

where *E*_*i*_′ and *AF*_*i*_ are normalized energy moment and amplitude factor (AF) for the *i*th IMF order, respectively. It should be noted that these features are selected based on the studied dataset; however, the feature selection practice for all similar datasets is the same. It means the features with highest FCF value should be selected for the input of any machine learning method.

In Table 7 a feature vector as a sample is depicted. It can be seen from the table that the input vector is composed of nine features. Although the output layer of the neural network contains two conditions (i.e., healthy and faulty), it is worth noting that the faulty condition encompasses three different faults. Since the data provided consist of two conditions, inevitably two output conditions are chosen for the neural network. The trend of fault feature vectors is constructed to detect faults individually. However, in this paper, because of the limitation of data, faults are detected simultaneously in one condition label.

The article "Intelligent Monitoring System Based on Noise-Assisted Multivariate Empirical Mode Decomposition Feature Extraction and Neural Networks" was published in 2022. Journal: Comput Intell Neurosci.

### 5.2. The Design Neural Network for the System

The main step in designing a neural network is to train the network based on the training samples. As mentioned earlier, the feature vectors in the input layer contain nine components. The number of nodes in the output layer is considered to be 2, corresponding to two conditions of system. 100 feature vectors are constructed for each system condition. 80% of data are considered as the training data and 20% as the testing data. In this study, a three-layer neural network is constructed for the intelligent fault diagnosis procedure. Therefore, according to (17) and network training conditions, the number of hidden layer nodes (*k*) is 18–26. In this study, *k*=18, since the differences between the output errors for the different values of *k* are in the same order (1e -5) while the learning rate is 0.001. The training function is TRAINLM to update the weight and bias values based on the Levenberg–Marquardt optimization method, and the activation function between the hidden layer and output layer is Sigmoid function. Note that the setting is similar for all experiments and all experiments have been done using MATLAB platform. Diagnosis rate for both training data and test data is 100%. This shows that the features and the network configuration are successfully selected.

## 6. Conclusion

In this paper, the MEMD algorithm is applied for extracting features from rotating machinery. To investigate the capacity of the proposed method, vibration signals from a wind turbine gearbox system as a rotating machinery system are utilized. When the rotating system is complex and consists of many faults, multiple sensors are exploited to obtain comprehensive information from the system. MEMD algorithm has the advantage of dealing with multivariate signals simultaneously. Usually, when the system is nonstationary and there are nonlinearity and multiple faults, using traditional features may be abortive. Features derived from the MEMD algorithm are based on the time and frequency domain, which compensate for the problem of using traditional features. To validate the effectiveness of the proposed features, a discrimination criterion is introduced. This criterion is based on the relativity of features to the fault classes.

The basic MEMD algorithm is sensitive to noise. In this study, an extension of MEMD called NA MEMD is implemented on multivariate signals to overcome the noise sensitivity of MEMD. MEMD algorithm decomposes signals into some signals named IMFs. Some of these IMFs are spurious and need to be eliminated from the calculation. A correlation factor is introduced to achieve this purpose. With the help of this factor, the number of redundant features is reduced. Two types of features are extracted from the IMFs. From the point of view of time-domain analysis, the energy moment of IMFs is a suitable feature, since it contains the time characteristics of signals. Therefore, this can be helpful when the signal is nonstationary. The other feature is in the frequency domain, and it relates to the amplitude of frequency spectrum in the characteristic frequencies. Because each IMF order encompasses a small frequency range, frequency analysis of IMFs is an effective way of highlighting characteristics.

The article "Intelligent Monitoring System Based on Noise-Assisted Multivariate Empirical Mode Decomposition Feature Extraction and Neural Networks" was published in 2022. Journal: Comput Intell Neurosci.

Based on the results, designing a neural network using the proposed features yields acceptable output results. The network is successfully trained using the training data, and the diagnostic rate is 100% not only for the training data, but also for the test data. It should be mentioned that the proposed algorithm is applied to real experimental data; however, by increasing the number of classes, the performance may decrease.

It should be noted that intelligent feature extraction using the proposed NA-MEMD method provides comprehensive information on the health status of the system. The proposed methodology gives higher explainability of the features compared to other similar methods. However, recently, deep learning-based methods have been successfully implemented in industrial datasets to automatically extract features. In spite of the effectiveness of these methods, they require high computation resources compared with the proposed method.

## Figures and Tables

**Figure 1:** Decomposition results by using NA-MEMD on the synthetic multivariate signal.

**Figure 2:** A typical BP neural network.

**Figure 3:** Intelligent fault detection flowchart.

**Figure 4:** Wind turbine planetary gearbox system (courtesy of NREL).

**Figure 5:** The characteristic frequency of the gearbox.

**Figure 6:** Decomposition results by using NA-MEMD on the synthetic multivariate signal.

**Table 1:** Traditional feature set parameters.

Time-domain features		Frequency-domain features	
Root mean square	$pt_{1}=\sqrt{\left(1/N\right)\sum_{n=1}^{N}x_{n}^{2}}$	Frequency barycenter	*pf*_1_=(∑_*k*=1_^*K*^*f*_*k*_*s*_*k*_/∑_*k*=1_^*K*^*s*_*k*_)
Peak	*pt*_2_=max(|*x*_*n*_|)	Root mean square frequency	$pf_{2}=\sqrt{\left(\sum_{k=1}^{K}f_{k}^{2}s_{k}/\sum_{k=1}^{K}s_{k}\right)}$
Square mean root	$pt_{3}={\left(\left(1/N\right)\sum_{n=1}^{N}\sqrt{\left|x_{n}\right|}\right)}^{2}$	Standard deviation frequency	$pf_{3}=\sqrt{\left(\sum_{k=1}^{K}{\left(f_{k}-pf_{1}\right)}^{2}s_{k}/\sum_{k=1}^{K}s_{k}\right)}$
Absolute mean	*pt*_4_=(1/*N*)∑_*n*=1_^*N*^(|*x*_*n*_|)	Frequency spectrum mean	*pf*_4_=(1/*N*)∑_*k*=1_^*K*^*s*_*k*_
Kurtosis	*pt*_5_=(1/*N*)∑_*n*=1_^*N*^*x*_*n*_^4^	Frequency spectrum deviation	*pf*_5_=(1/*K* − 1)∑_*k*=1_^*K*^(*s*_*k*_ − *pf*_4_)^2^
Crest factor	*pt*_6_=(*pt*_1_)/(*pt*_2_)	Frequency spectrum entropy	$pf_{6}=-\sum_{k=1}^{K}\left(s_{k}/Kpf_{4}\right)\log\left(\left(s_{k}\right)/Kpf_{4}\right)$

The article "Intelligent Monitoring System Based on Noise-Assisted Multivariate Empirical Mode Decomposition Feature Extraction and Neural Networks" was published in 2022. Journal: Comput Intell Neurosci.

**Table 2:** Fault correlation factor for synthetic multivariate signal.

IMF order	1	2	3	4	5	6	7	8	9	10
FCF	0.2131	0.1965	0.6491	0.4125	0.6600	0.0224	0.0208	0.0366	0.0376	0.0191

**Table 3:** Dimensions and mechanical details of the gear element [48].

Gear Elements	No. of teeth	Mate teeth	Root diameter (mm)	Helix angle	Face width (mm)	Ratio
Ring gear	99	39	1047	7.5 L	230	
Planet gear	39	99	372	7.5 L	227.5	
Sun gear	21	39	186	7.5 R	220	5.71
Intermediate gear	82	23	678	14 R	170	
Intermediate pinion	23	82	174	14 L	186	3.57
High-speed gear	88	22	440	14 L	110	
High-speed pinion	22	88	100	14 R	120	4.0
					Overall:	81.49

**Table 4:** Characteristic frequencies formulations.

Component	Characteristic frequency	Formulation
Fixed-axis gearbox	Meshing frequency	*f*_*m*_=*f*_1_*N*_1_=*f*_2_*N*_2_

Planetary stage	Planet frequency [49]	*f*_*p*_=((*N*_*p*_ − *N*_*R*_)*N*_*s*_/(*N*_*R*_+*N*_*s*_)*N*_*p*_)*f*_*s*_
	Carrier frequency [49]	*f*_*c*_=(*N*_*s*_/*N*_*R*_+*N*_*s*_)*f*_*s*_
	Meshing frequency [49]	*f*_*m*−*p*_=(*f*_*s*_ − *f*_*c*_)*N*_*s*_=(*N*_*R*_*N*_*S*_/*N*_*R*_+*N*_*S*_)*f*_*s*_

Bearing	Ball pass frequency, outer race [50]	*BPFO*=(*nf*_*r*_/2){1 − (*d*/*D*)cos*ϕ*}
	Ball pass frequency, inner race [50]	*BPFI*=(*nf*_*r*_/2){1+(*d*/*D*)cos*ϕ*}
	Fundamental train frequency (cage speed) [50]	*FTF*=(*f*_*r*_/2){1 − *d*/*D*cos*ϕ*}
	Ball (roller) spin frequency [50]	*BSF*(*RSF*)=(*D*/2 *d*){1 − ((*d*/*D*)cos*ϕ*)}^2^

**Table 5:** Correlation coefficient factor for each IMF.

IMF order/FCF																			
1	2	3	4	5	6	7	8	9	10	11	12	13	14	15	16	17	18	19	20
0.1084	0.2254	0.6318	0.8279	0.4050	0.4152	0.3245	0.3014	0.0214	0.0212	0.0368	0.0039	0.0006	0.0001	0.0002	0.0002	0.0001	0.0001	0.0001	0.0002

**Table 6:** Discrimination criterion for the proposed features.

Feature	*AF*_6_	*AF*_8_	*E*_3_′	*E*_4_′	*pt*_1_	*E*_5_′	*E*_6_′	*E*_7_′	*AF*_11_	*E*_8_′	*pt*_*i*_, *pf*_1_, *pf*_*i*_^*∗*^
J criterion's value	1.932	1.812	1.720	1.600	1.541	1.021	0.952	0.741	0.603	0.402	≤0.1

**Table 7:** Neural network input and output vector.

Feature vector	System condition
[0.0826, 07469,0.0877, 0.0200, 0.0261, 0.0367, 0.0477, 0.0409, 0.0535]	Healthy
[0.2125, 0.5985, 0.0347, 0.0664, 0.0052, 0.0826, 0.5308, 0.7147, 0.0659]	Faulty

The article "Intelligent Monitoring System Based on Noise-Assisted Multivariate Empirical Mode Decomposition Feature Extraction and Neural Networks" was published in 2022. Journal: Comput Intell Neurosci.

## Data Availability

The NREL wind turbine data used to support the findings of this study are included within the article.
